# Efficacy and Safety Analysis of Multislice Spiral CT-Guided Transthoracic Lung Biopsy in the Diagnosis of Pulmonary Nodules of Different Sizes

**DOI:** 10.1155/2022/8192832

**Published:** 2022-08-25

**Authors:** Huitong Liu, Xiao Yao, Bingqiang Xu, Wei Zhang, Yu Lei, Xiaolong Chen

**Affiliations:** Shaanxi Provincial People's Hospital, Xi'an, Shaanxi Province 710068, China

## Abstract

**Objective:**

This study is aimed at investigating the efficacy and safety of multislice spiral CT-guided transthoracic lung biopsy in the diagnosis of pulmonary nodules of different sizes.

**Methods:**

Data of 78 patients with pulmonary nodules who underwent CT-guided transthoracic lung biopsy in our hospital from January 2020 to December 2021 were retrospectively analyzed, and they were divided into the small nodules group (*n* = 12), medium nodules group (*n* = 35), and large nodules group (*n* = 31) according to the diameter of pulmonary nodules. The results of puncture biopsy and final diagnosis of pulmonary nodules of different sizes were compared. The incidence of complications in patients with pulmonary nodules of different sizes was compared. Univariate analysis was used to compare the incidence of complications in 78 patients. Logistic multiple regression analysis was used to analyze the independent risk factors of pneumothorax in patients with pulmonary nodule puncture. Logistic multiple regression analysis was used to analyze the independent risk factors of pulmonary hemorrhage in patients with pulmonary nodule puncture.

**Results:**

The diagnostic accuracy, sensitivity, and specificity were 83.33%, 100.00%, and 77.78% in small nodules group. The diagnostic accuracy, sensitivity, and specificity of medium nodules group were 85.71%, 100.00%, and 73.68%, respectively. The diagnostic accuracy, sensitivity, and specificity of large nodules group were 93.55%, 100.00%, and 33.33%, respectively. There was no significant difference in the incidence of pneumothorax among the three groups (*P* > 0.05). The incidence of pulmonary hemorrhage in small nodule group was higher than that in the medium nodule group and large nodule group, and the difference was statistically significant (*P* < 0.05). There was no significant difference in the incidence of total complications among the three groups (*P* > 0.05). There were statistically significant differences in clinical data such as the needle tract length, the puncture position, and the distance of the puncture needle passing through the lung tissue in patients with or without pneumothorax (*P* < 0.05). There were statistically significant differences in needle tract length, distance of puncture needle passing through lung tissue, and size of pulmonary nodules in patients with or without pulmonary hemorrhage (*P* > 0.05). Logistic multivariate analysis showed that needle tract length ≤ 50 mm, lateral decubitus position, and the distance of puncture needle passing through lung tissue ≥ 14 mm were independent risk factors for pneumothorax after puncture in patients with pulmonary nodules (*P* < 0.05). The needle tract length > 50 mm, the distance of puncture needle passing through lung tissue ≥ 14 mm, and small nodules (pulmonary nodules diameter ≤ 10 mm) were independent risk factors for pulmonary hemorrhage after puncture in patients with pulmonary nodules (*P* < 0.05).

**Conclusion:**

Multislice spiral CT-guided transthoracic lung biopsy is effective in diagnosing pulmonary nodules of different sizes.

## 1. Introduction

Pulmonary nodules refer to lesions with a diameter of ≤30 mm in the lungs. The lung nodules are round or quasiround in shape and surrounded by air-filled lung tissue. According to CT imaging morphology, pulmonary nodules can be divided into solid nodules, partially solid nodules, and ground glass nodules [1]. The incidence of pulmonary nodules is 35.5%, of which pulmonary nodules diagnosed as lung cancer account for 0.54%, respectively; the incidence of pulmonary nodules among people who smoke more than 30 packs per year is 25.9%, of which pulmonary nodules diagnosed as lung cancer accounted for 1.1% [2]. The etiology of pulmonary nodules is complex and diverse, including infectious factors, tumor factors, and pulmonary infectious factors [3, 4]. It is reported that pulmonary nodules with diameter < 5 mm have a 0.4% probability of developing into carcinoma in situ, pulmonary nodules with diameter of 5-10 mm have a 1.3% probability of developing into malignancy, pulmonary nodules with diameter of 10-20 mm have a 50% probability of developing into malignancy, and pulmonary nodules with diameter > 20 mm have an 87.5% probability of developing into malignancy. Pulmonary nodules of different sizes have different probability of developing into malignancy, so early diagnosis of pulmonary nodules is very important [5]. Lung biopsy has high diagnostic accuracy and can also judge the differentiation degree of malignant tumor, which can effectively guide clinical treatment. Transthoracic lung biopsy was first applied to the microbiological diagnosis of patients with lung infection in 1882, and the first lung cancer biopsy was performed in 1886. Later, it was gradually developed to use ultrasound, CT, etc. for lung biopsy. CT is the most widely used guidance method in clinical practice, with high soft tissue contrast ability and spatial resolution. CT-guided puncture biopsy of pulmonary nodules also has high diagnostic accuracy and safety [6–9]. Multislice spiral CT refers to an imaging system with a multirow detector structure and a single exposure of the tube, which can simultaneously obtain data from multiple slices of images [10]. Compared with traditional CT-guided lung biopsy, multislice CT-guided lung biopsy has the advantages of fast scanning speed and shorter scanning time. In addition, the repeated scanning procedure of multislice spiral CT-guided lung biopsy can make the guidance easier to operate [11]. The purpose of this study was to investigate the diagnostic efficacy of multislice spiral CT-guided transthoracic lung biopsy for pulmonary nodules of different sizes. The report is as follows.

## 2. Materials and Methods

### 2.1. General Information

Data of 78 patients with pulmonary nodules who underwent multislice spiral CT-guided transthoracic lung biopsy in our hospital from January 2020 to December 2021 were retrospectively analyzed. There were 55 males and 23 females, aged from 20 to 78 years old, with an average age of 49.55 ± 5.63 years old; 12 cases with pulmonary nodule diameter ≤ 10 mm were divided into small nodule group; 35 cases with pulmonary nodule diameter ≤ 20 mm were divided into middle nodule group; 31 cases with pulmonary nodule diameter > 20 mm and ≤ 30 mm were divided into large nodule group. This study was approved by the hospital ethics committee.

### 2.2. Inclusion Criteria

Inclusion criteria are as follows: (1) 0 mm < pulmonary nodule diameter ≤ 30 mm; (2) age ≥ 18 years old; (3) no contraindications for CT-guided transthoracic lung biopsy; (4) complete clinical and imaging data; (5) the chest CT examination showed pulmonary nodules; and (6) patients volunteered to participate in this study.

### 2.3. Exclusion Criteria

Exclusion criteria are as follows: (1) patients with intrapulmonary vascular disease; (2) patients with pulmonary fibrosis, pulmonary hypertension, and severe emphysema; (3) patients with severe bleeding tendency or coagulation dysfunction; (4) patients who cannot cooperate with breathing; (5) the heart and blood vessels cannot be avoided during the puncture of the lesion; (6) patients with lung bullae lesions in puncture approach; (7) patients with severe pulmonary infection; and (8) there is skin infection at the site to be punctured.

### 2.4. Methods

#### 2.4.1. Operation Instrument

Canon Aquilion ONE 640CT was used, and the puncture needle was a shotgun-cut biopsy needle. The imaging data of the patients were carefully observed before surgery, and the lateral, supine, and prone positions were adopted according to the size and location of the lung nodules. First, local scan of the lesion was carried out with a layer thickness of 2.7 mm. The best puncture point was selected by CT positioning ruler, and the distance between the puncture point and the edge and center of the lesion as well as the puncture direction and angle were measured. Routine disinfection and draping were performed, local anesthesia was performed, anesthesia needle was injected 1~2 cm in accordance with the expected puncture direction and angle, the puncture biopsy scanning procedure was used to scan to verify whether there was any error in puncture point, puncture direction, and angle, and the scan could be performed again after appropriate adjustment. The patient was told to keep calm breathing and hold his breath, and after confirmation, the shotgun-cut biopsy needle was used to rapidly puncture the lung lesions of the patient. After reaching the expected depth, the scan was carried out to confirm that the needle tip was in the patient's lesion. Then the patient was told to hold his breath, the lesion tissue was cut, the needle was removed quickly, and the tissue specimen was fixed with formalin and then sent for examination. If the pathologist is not satisfied, the needle biopsy should be performed again and the liquefaction necrotic area should be avoided. After surgery, the puncture site was pressed for 2~3 minutes, external dressing was applied, and then the lungs were scanned to observe whether the patient had bleeding, pneumothorax, and other complications.

### 2.5. Judgment Criteria for Puncture Results

(1) If the biopsy tissue is normal lung tissue and diaphragmatic muscle according to pathological results, it is regarded as failure of sampling. (2) If the pathological examination result of biopsy tissue is malignant tumor, the pathological diagnosis is definite. (3) If the pathological examination result of biopsy tissue is benign and confirmed by surgery, or the lesions disappear, shrink, and stabilize for more than half a year after treatment, it is regarded as correct pathological diagnosis. The accuracy of puncture biopsy can be obtained by comparing the final clinical examination results with the results of needle biopsy.

### 2.6. Observation Indicators

Observation indicators are as follows: (1) general information of all patients; (2) comparison of puncture biopsy and final diagnosis results of pulmonary nodules of different sizes; (3) comparison of the incidence of complications among patients with pulmonary nodules of different sizes; (4) univariate analysis of the incidence of complications in all patients; (5) logistic multiple regression analysis was used to analyze the independent risk factors of pneumothorax in patients with pulmonary nodule puncture; and (6) logistic multiple regression analysis was used to analyze the independent risk factors of pulmonary hemorrhage in patients with pulmonary nodule puncture.

### 2.7. Statistical Methods

All data in this study were input into Excel by two persons without communication and analyzed and processed by the SPSS24.0 statistical software. The measurement data were expressed as mean ± SD (*x̅*±*s*). When the data were in line with normal distribution and the variance was uniform, the *t* test was adopted, and one-way ANOVA was used comparison among multiple groups. Counting data were described by *n* and %, and disordered classification data were compared by the *χ*^2^ test or Fisher's exact probability method. Multivariate analysis was performed by the logistic regression model. All were two-sided tests, and *P* < 0.05 was considered statistically significant.

## 3. Results

### 3.1. General Information of Patients

The general information of all patients is shown in Table 1.

### 3.2. Comparison of Puncture Biopsy and Final Diagnosis Results of Pulmonary Nodules of Different Sizes

In the small nodules group, the diagnostic accuracy, sensitivity, and specificity were 83.33%, 100.00%, and 77.78%, respectively, the positive prediction rate was 60.00%, the negative prediction rate was 81.82%. In the medium nodules group, the diagnostic accuracy, sensitivity, and specificity were 85.71%, 100.00%, and 73.68%, respectively, the positive prediction rate was 76.19%, and the negative prediction rate was 79.17%. In the large nodules group, the diagnostic accuracy, sensitivity, and specificity were 93.55%, 100.00%, and 33.33%, respectively, the positive prediction rate was 93.55%, and the negative prediction rate was 60.00% (see Tables 2 and 3 and Figure 1).

### 3.3. Comparison of Complications among the Three Groups

There was no significant difference in the incidence of pneumothorax among the three groups (*P* > 0.05); the incidence of pulmonary hemorrhage in the small nodules group was higher than that in the middle nodules group and the large nodules group, and the difference was statistically significant (*P* < 0.05). There was no significant difference in the total incidence of complications among the three group (*P* > 0.05) (see Table 4).

### 3.4. Univariate Analysis of Complications in 78 Patients

There were statistically significant differences in clinical data such as the needle tract length, the puncture position, and the distance of the puncture needle passing through the lung tissue in patients with or without pneumothorax (*P* < 0.05). There were statistically significant differences in needle tract length, distance of puncture needle passing through lung tissue, and size of pulmonary nodules in patients with or without pulmonary hemorrhage (*P* < 0.05), as shown in Table 5.

### 3.5. Logistic Multivariate Regression Analysis of the Incidence of Pneumothorax in 78 Patients

Factors with statistically significant differences in the above univariate analysis of pneumothorax, including needle track length, puncture position, and distance of puncture needle passing through lung tissue, were included in the logistic regression analysis and assigned (needle track length > 50 mm = 1, ≤50 mm = 0; puncture position: supine position = 2, prone position = 1, and lateral position = 0; the distance of the puncture needle passing through the lung tissue < 14 mm = 1, ≥14 mm = 0). Logistic multivariate analysis showed that needle length ≤ 50 mm, lateral position, and the distance of puncture needle passing through lung tissue ≥ 14 mm were independent risk factors for pneumothorax after puncture in patients with pulmonary nodules (*P* < 0.05), as shown in Table 6.

### 3.6. Logistic Multivariate Regression Analysis of the Incidence of Pulmonary Hemorrhage in 78 Patients

Factors with statistically significant differences in the above univariate analysis of pulmonary hemorrhage, including needle track length, distance of puncture needle passing through lung tissue, and the size of the pulmonary nodule, were included in Logistic regression analysis and assigned (needle track length ≤ 50 mm = 1, >50 mm = 0; distance of puncture needle passing through lung tissue < 14 mm = 1, ≥14 mm = 0; large nodule (20 mm < pulmonary nodule diameter ≤ 30 mm) = 2, medium nodule (10 mm < pulmonary nodule diameter ≤ 20 mm) = 1, and small nodules (pulmonary nodule diameter ≤ 10 mm) = 0). Logistic multivariate analysis results showed that the needle tract length > 50 mm, the distance of the puncture needle passing through the lung tissue ≥ 14 mm, and the small nodule (pulmonary nodule diameter ≤ 10 mm) were independent risk factor for pulmonary hemorrhage after puncture in patients with pulmonary nodules (*P* < 0.05) (see Table 7).

## 4. Discussion

Lung biopsy, open lung biopsy, thoracoscopy biopsy, and fiberoptic bronchoscopy biopsy can all obtain histopathological specimens of lung lesions, but open lung biopsy and thoracoscopic biopsy are more traumatic to the body, and their application is limited in elderly patients and patients with cardiopulmonary dysfunction [12–14]. Lung puncture biopsy has little trauma, low cost, and less pain to patients. Some patients do not need to be hospitalized after puncture and can live a normal life the next day. In addition, CT scan has good contrast and resolution, which can clearly display the morphology, size, and adjacent important structure of lesions and can display small lesions beside the mediastinum, behind the heart shadow, and beside the spine [15, 16]. It has been reported that the accuracy of CT-guided lung biopsy in the diagnosis of benign lesions is >80% and that of malignant lesions is >90% [17]. In this study, the diagnostic efficiency of multislice spiral CT for pulmonary nodules of different sizes was observed. The results showed that the diagnostic accuracy of the small nodule group was 83.33%, the sensitivity was 100.00%, the specificity was 77.78%, the positive predictive rate was 60.00%, and the negative predictive rate was 81.82%. In the middle nodule group, the diagnostic accuracy was 85.71%, the sensitivity was 100.00%, the specificity was 73.68%, the positive predictive rate was 76.19%, and the negative predictive rate was 79.17%. In the large nodule group, the diagnostic accuracy was 93.55%, sensitivity was 100.00%, specificity was 33.33%, the positive predictive rate was 93.33%, and negative predictive rate 60.00%. Multislice spiral CT-guided lung biopsy has the highest diagnostic accuracy for diagnosing large nodules (20 mm < pulmonary nodule diameter ≤ 30 mm). The sensitivity of multislice spiral CT-guided lung biopsy in the diagnosis of lung nodules of different sizes was up to 100.00%, indicating that multislice spiral CT-guided lung biopsy is an effective method for the diagnosis of lung cancer.

Common complications of transthoracic lung biopsy include pneumothorax, pulmonary hemorrhage, and hemoptysis, and the rare serious complications include air embolism and tumor needle passage metastasis [18, 19]. In this study, complications of multislice spiral CT-guided lung biopsy were observed, and the results showed that there was no statistical significance in the incidence of pneumothorax in groups of different sizes of pulmonary nodules. According to relevant reports, the incidence of pneumothorax of CT-guided transthoracic lung biopsy is 15.4%~42.0%, only 4.3%~7.3% patients need thoracic catheter drainage, and the incidence of hemoptysis is 0.5%~14.4%, most of which do not need intervention [20, 21]. The common risk factors of pneumothorax include long puncture path, multiple crossing of pleura, and small lesion [22, 23]. In this study, univariate and multivariate analyses were conducted on the risk factors for pneumothorax and pulmonary hemorrhage, and it was found that needle tract length ≤ 50 mm, lateral position, and the distance of puncture needle passing through lung tissue ≥ 14 mm were independent risk factors for pneumothorax after puncture in patients with pulmonary nodules. The results of this study suggest that when the puncture needle tract is ≤50 mm, the risk of pneumothorax increases, which is contrary to the results of previous studies [24, 25]. The reason may be that the shorter the puncture needle tract, the gas in the lung will pass through the needle in a short time, thus causing pneumothorax. In this study, the poor postural stability of patients in lateral position also easily led to an increase in the incidence of pneumothorax after puncture. In this study, the distance of puncture needle passing through the lung tissue is closely related to the occurrence of pneumothorax, which is manifested as the greater the distance of puncture needle passing through the lung tissue, the more likely pneumothorax will occur. This may be because when people breathe, there is sliding between visceral pleura and parietal pleura, and indirect friction can be formed when the needle is fixed with chest wall muscle layer, which can lead to pneumothorax. The longer the distance of puncture needle passing through the lung tissue, the more obvious the friction effect is. Therefore, the needle tract length ≤ 50 mm, lateral position, and the distance of puncture needle passing through the lung tissue ≥ 14 mm are independent risk factors for pneumothorax in patients with pulmonary nodules after puncture. It is suggested that full attention should be paid to patients with needle tract length ≤ 50 mm, lateral position, and the distance of puncture needle passing through lung tissue ≥ 14 mm to prevent pneumothorax in time.

In this study, logistic multivariate analysis showed that the needle tract length > 50 mm, the distance of the puncture needle passing through the lung tissue ≥ 14 mm, and small nodules (pulmonary nodule diameter ≤ 10 mm) were independent risk factors for pulmonary hemorrhage after puncture in patients with pulmonary nodules (*P* < 0.05). It was reported that the incidence of pulmonary hemorrhage after puncture was 16%-33%. In this study, the incidence of pulmonary hemorrhage was higher in the small nodules group, and the overall incidence of pulmonary hemorrhage was consistent with the results of previous studies [26–28]. This study found that the longer the needle track, the easier it is to cause pulmonary hemorrhage, which is consistent with previous research results [29, 30]. The longer the needle track is, the more it passes through the lung tissue, which can lead to injury and bleeding. Therefore, the needle track length > 50 mm and the distance of the needle passing through the lung tissue ≥ 14 mm are closely related to pulmonary hemorrhage. In this study, the pulmonary nodule diameter ≤ 10 mm was an independent risk factor for pulmonary hemorrhage. This may be because when the lesion is small, the puncture process is greatly affected by breathing, and the needle needs to be adjusted several times during the puncture process, which is likely to cause pulmonary hemorrhage. In addition, if the lesion is small, normal tissue may be removed to obtain sufficient tissue specimens, resulting in increased bleeding rate. Therefore, prevention of pulmonary hemorrhage should be done well for patients with needle tract length > 50 mm, the distance of puncture needle passing through lung tissue ≥ 14 mm, and small nodules (lung nodules diameter ≤ 10 mm).

In conclusion, multislice spiral CT-guided lung biopsy has high accuracy in diagnosing pulmonary nodules, and the complication rates of pneumothorax and pulmonary hemorrhage are consistent with previous research results [31], which has clinical application value. However, in this study, the sample size is small and the classification method of nodule size is different from that of most literatures. In future research, the sample size of the study will be further expanded and the grouping of nodule size will be improved, to provide more scientifically rigorous clinical research results in the diagnosis of pulmonary nodules by multislice spiral CT-guided lung biopsy.

## Figures and Tables

**Figure 1:** A 54-year-old male patient, with a nodule in the left lower lobe found by physical examination before 2 weeks. (a) A solid nodule in the lateral basal segment of the left lower lobe, with a diameter of about 1.3 cm (indicated by the arrow). (b) The needle was obliquely inserted from the adjacent intercostal space, avoiding the scapula. (c) After needle extraction, there was a small amount of bleeding and pneumothorax (indicated by the arrow), and the pneumothorax were absorbed after observation. (d) The surgical pathological results were the same after puncture, and invasive adenocarcinoma was considered (×100, HE staining).

**Table 1:** General information of patients (cases (%)).

Item	Composition ratio
Lung nodule location	
Right upper lobe	29 (37.18)
Right middle lobe	9 (11.54)
Right lower lobe	17 (21.79)
Left upper lobe	12 (15.38)
Left lower lobe	11 (14.10)
Previous tumor history	
Yes	3 (3.85)
No	75 (96.15)
Smoking history	
Yes	41 (52.56)
No	37 (47.44)
Puncture position	
Supine position	25 (32.05)
Prone position	44 (56.41)
Lateral position	9 (11.54)

**Table 2:** Comparison of puncture biopsy and final diagnosis results of pulmonary nodules of different sizes (cases (%)).

Group	Biopsy diagnosis result		Final diagnosis result	
	Benign	Malignant	Benign	Malignant
Small nodules group (*n* = 12)	7 (58.33)	5 (41.67)	9 (75.00)	3 (25.00)
Medium nodules group (*n* = 35)	14 (40.00)	21 (60.00)	19 (54.29)	16 (45.71)
Large nodules group (*n* = 31)	1 (3.23)	30 (96.77)	3 (9.68)	28 (90.32)
Total	22	56	31	47

**Table 3:** Comparison of diagnostic accuracy, sensitivity, specificity, positive predictive rate, and negative predictive rate of puncture biopsy among the three groups (%).

Group	Accuracy	Sensitivity	Specificity	Positive predictive rate	Negative predictive rate
Small nodules group (*n* = 12)	83.33	100.00	77.78	60.00	81.82
Medium nodules group (*n* = 35)	85.71	100.00	73.68	76.19	79.17
Large nodules group (*n* = 31)	93.55	100.00	33.33	93.33	60.00

**Table 4:** Comparison of the incidence of complications among the three groups (cases (%)).

Group	Pneumothorax	Pulmonary hemorrhage	Total complication rate
Small nodules group (*n* = 12)	2 (16.67)	7 (58.33)	9 (75.00)
Medium nodules group (*n* = 35)	6 (17.14)	8 (22.86)	14 (40.00)
Large nodules group (*n* = 31)	7 (22.58)	5 (16.13)	12 (38.71)

**Table 5:** Univariate analysis of complications in 78 patients.

Item	Pneumothorax				Pulmonary hemorrhage			
	Yes (*n* = 15)	No (*n* = 63)	*t*/*χ*^2^ value	*P*/Fisher's exact probability value	Yes (*n* = 20)	No (*n* = 58)	*t*/*χ*^2^ value	*P* value
Age								
<60 years old (*n* = 29)	6 (20.69)	23 (79.31)	0.063	0.801	5 (17.24)	24 (82.76)	1.708	0.191
≥60 years old (*n* = 49)	9 (18.37)	40 (81.63)			15 (30.61)	34 (69.39)		
Gender								
Male (*n* = 55)	11 (20.00)	44 (80.00)	0.071	0.790	13 (23.64)	42 (76.36)	0.393	0.531
Female (*n* = 23)	4 (17.39)	19 (82.61)			7 (30.43)	16 (69.57)		
Nodule density (cases)								
Solid (*n* = 67)	14 (20.90)	53 (79.10)	0.848	0.357	16 (23.88)	51 (76.12)	0.772	0.380
Nonsolid (*n* = 11)	1 (9.09)	10 (90.91)			4 (36.36)	7 (63.64)		
Needle track length								
≤50 mm (*n* = 17)	7 (41.18)	10 (58.82)	6.740	0.009	1 (5.88)	16 (94.12)	4.451	0.035
>50 mm (*n* = 61)	8 (13.11)	53 (86.89)			19 (31.15)	42 (68.85)		
Puncture lung lobe								
Right upper lobe (*n* = 29)	4 (13.79)	25 (86.21)	1.315	0.859	7 (24.14)	22 (75.86)	3.338	0.503
Right middle lobe (*n* = 9)	2 (22.22)	7 (77.78)			1 (11.11)	8 (88.89)		
Right lower lobe (*n* = 17)	4 (23.53)	13 (76.47)			4 (23.53)	13 (76.47)		
Left upper lobe (*n* = 12)	2 (16.67)	10 (83.33)			3 (25.00)	9 (75.00)		
Left lower lobe (*n* = 11)	3 (27.27)	8 (72.73)			5 (45.45)	6 (54.55)		
Smoking history								
Yes (*n* = 41)	8 (19.51)	33 (80.49)	0.004	0.947	11 (26.83)	30 (73.17)	0.064	0.800
No (*n* = 37)	7 (18.92)	30 (81.08)			9 (24.32)	28 (75.68)		
Puncture position								
Supine position (*n* = 25)	2 (8.00)	23 (92.00)	—	0.001	7 (28.00)	18 (72.00)	1.131	0.568
Prone position (*n* = 44)	7 (15.91)	37 (84.09)			12 (27.27)	32 (72.73)		
Lateral position (*n* = 9)	6 (66.67)	3 (33.33)			1 (11.11)	8 (88.89)		
Number of punctures								
1~3 times (*n* = 35)	7 (20.00)	28 (80.00)	0.024	0.876	10 (28.57)	25 (71.43)	0.286	0.593
≥4 times (*n* = 43)	8 (18.60)	35 (81.40)			10 (23.26)	33 (76.74)		
Distance of puncture needle passing through lung tissue (mm)	22.15 ± 2.55	13.56 ± 2.35	12.520	<0.001	24.19 ± 5.68	12.68 ± 3.25	11.101	<0.001

**Table 6:** Logistic multivariate regression analysis of the incidence of pneumothorax in 78 patients.

Factor	*β*	SE	Wald *χ*^2^	OR	95% CI	*P*
Needle track length ≤ 50 mm	0.521	0.225	5.362	1.684	1.083~2.617	0.021
Lateral position	0.355	0.134	7.019	1.426	1.097~1.855	0.008
Distance of the puncture needle passing through the lung tissue ≥ 14 mm	1.526	0.554	7.587	4.600	1.553~13.624	0.006

**Table 7:** Logistic multivariate regression analysis of the incidence of pulmonary hemorrhage in 78 patients.

Factor	*β*	SE	Wald *χ*^2^	OR	95% CI	*P*
Needle track length > 50 mm	1.159	0.452	6.575	3.187	1.314~7.729	0.011
Distance of puncture needle passing through lung tissue ≥ 14 mm	1.594	0.686	5.399	4.923	1.283~18.889	0.021
Small nodules	1.403	0.545	6.627	4.067	1.398~11.837	0.010

## Data Availability

The labeled dataset used to support the findings of this study are available from the corresponding author upon request.
